The article "Toll-like receptor 9 (TLR9) gene deletion-mediated fracture healing in type II diabetic osteoporosis associates with inhibition of the nuclear factor-kappa B (NF-κB) signaling pathway" was retracted in 2026. Reasons: concerns about the data; concerns about the results or conclusions.

# Toll-like receptor 9 (TLR9) gene deletion-mediated fracture healing in type II diabetic osteoporosis associates with inhibition of the nuclear factor-kappa B (NF-κB) signaling pathway

**DOI:** 10.1080/21655979.2022.2063663

**Published:** 2022-06-15

**Authors:** Jiakai Han, Qian Zheng, Yongxia Cheng, Yong Liu, Yuxin Bai, Bin Yan, Sufen Guo, Jianbo Yu, Xinxin Li, Chong Wang

**Affiliations:** a Endocrinology Department, Huaihe Hospital of Henan University, Kaifeng, PR, China; b Endocrinology Department, Yan’an Hospital of Kunming Medical University, Kunming, PR, China; c Pathology Diagnosis Center, The HongQi Hospital, The First Clinical Medical School of Mudanjiang Medical College, Mudanjiang, PR, China; d Platform Management Division, Scientific Research Division of Mudanjiang Medical College, Mudanjiang, PR, China; e Ultrasound Department, Second Hospital of Mudanjiang Medical College, Mudanjiang, PR, China

**Keywords:** TLR9 knockout, NF-κB signaling pathway, type II diabetic osteoporosis, fracture healing

## Abstract

Diabetes is characterized by increased fracture risk. Evidence from *in vivo* studies is lacking for anti-fracture strategies in diabetes. Our microarray analyses predicted association of Toll-like receptor 9 (TLR9) with both diabetes and osteoporosis, which was the focus of this work in a murine model of type II diabetic osteoporosis (T2DOP). A T2DOP model with fracture was established in TLR9 knockout (TLR9^−/−^) mice, which were then treated with the NF-κB signaling pathway inhibitor (PDTC) and activator (TNF-α). The obtained data suggested that TLR9 knockout augmented regeneration of bone tissues and cartilage area in the callus, and diminished fibrous tissues in T2DOP mice. Moreover, TLR9 depletion significantly affected bone mineral density (BMD), bone volume/tissue volume (BV/TV), connectivity density, trabecular number, trabecular separation and trabecular thickness, thus promoting fracture recovery. Bone morphology and structure were also improved in response to TLR9 depletion in T2DOP mice. TLR9 depletion inactivated NF-κB signaling in T2DOP mice. PDTC was found to enhance fracture healing in T2DOP mice, while TNF-α negated this effect. Collectively, these data indicate that TLR9 depletion may hold anti-fracture properties, making it a potential therapeutic target for T2DOP.

**Abbreviations:** Diabetic osteoporosis (DOP); bone mineral density (BMD); Toll-like receptors (TLRs); type 2 diabetes (T2D); Toll-like receptor 9 (TLR9); nuclear factor-kappaB (NF-κB); streptozotocin (STZ); type 2 diabetic osteoporosis (T2DOP); Gene Expression Omnibus (GEO); Kyoto encyclopedia of genes and genomes (KEGG); pyrrolidine dithiocarbamate (PDTC); computed tomography (CT); Hematoxylin–eosin (HE); bone morphogenetic protein 7 (BMP7); analysis of variance (ANOVA);

The article "Toll-like receptor 9 (TLR9) gene deletion-mediated fracture healing in type II diabetic osteoporosis associates with inhibition of the nuclear factor-kappa B (NF-κB) signaling pathway" was retracted in 2026. Reasons: concerns about the data; concerns about the results or conclusions.

## Highlights

- TLR9 mediates NF-κB signaling pathway and affects T2DOP.
- Knockout of TLR9 promotes callus formation in the fracture of mice with T2DOP.
- Knockout of TLR9 inhibits NF-κB pathway to promote fracture healing in T2DOP.
- Knockout of TLR9 promotes callus formation in the fracture of mice with T2DOP.
- This study provides a new target for the diagnosis and treatment of T2DOP.

## 1. Introduction

It is known to us all that osteoporosis and diabetes are common diseases presenting significant associated morbidity and mortality [1]. Diabetic osteoporosis (DOP), as a prevalent complication of diabetes, presents a rising incidence over the past few decades [2], and can lead to increased fracture risk and impaired bone healing [3]. Management of the bone fractures has been complicated due to the poor bone quality, possibly leading to inadequate fixation strength and stability [4]. This systemic endocrine-metabolic osteopathy is characterized by reduction in bone mineral density (BMD) and destruction of bone microstructure [5]. An increasing number of scholars have been exploring the treatment for DOP. Silibinin was suggested to be potential for treatment of DOP [6]. Moreover, traditional Chinese medicine Bushen-Jianpi-Huoxue decoction has also been highlighted as a treatment strategy for DOP [7]. In spite of this context, further study on control of DOP is still urgent.

Toll-like receptors (TLRs) are identified as family members of conserved pattern recognition receptors [8] and function as an activator of inflammation and associated development of chronic degenerative disorders such as type 2 diabetes mellitus (T2D) [9]. Toll-like receptor 9 (TLR9), one of the important members of TLRs, is an innate immune receptor which recognizes microbial DNA [10]. A significant increase of the expression of TLR9 has been confirmed in rats following hip fracture [11]. Intriguingly, deficiency of TLR9 was found to enhance glucose tolerance, and improve insulin sensitivity of type 1 diabetes [12]. Notably, the TLR9/nuclear factor-kappaB (NF-κB) signaling pathway is responsible for hip fracture-induced lung injury [11]. It is noteworthy that degradation of TLR9 mediated by Triad3A contributes to suppressed activation of the NF-κB signaling pathway, thereby preventing the progression of cardiac hypertrophy [13]. Moreover, a previous study reported that TLR9 could induce the NF-κB signaling pathway in cancer-associated fibroblasts [14]. In addition, NF-κB transcription factor activation is critical for a wide range of processes such as immunity, inflammation, oxidative stress, cell development, growth and survival [15–17]. Of note, it was previously demonstrated that activation of the NF-κB signaling pathway is one of the leading causes of the occurrence of DOP [18]. Additionally, expression of NF-κB stimulated by receptor activator of nuclear factor (NF)-κB-ligand (RANKL) can be downregulated by silencing of MLN64, thus alleviating DOP in the streptozotocin (STZ)-induced mouse model [19].

The article "Toll-like receptor 9 (TLR9) gene deletion-mediated fracture healing in type II diabetic osteoporosis associates with inhibition of the nuclear factor-kappa B (NF-κB) signaling pathway" was retracted in 2026. Reasons: concerns about the data; concerns about the results or conclusions.

Considering the aforementioned reports, we speculated that TLR9 may activate the NF-κB signaling pathway and consequently participated in the fracture healing in type 2 diabetic osteoporosis (T2DOP). Hence, the main objective of this study was to determine if the aforementioned hypothesis was valid and to further elucidate the interactions between TLR9 and the NF-κB signaling pathway as well as the associated mechanisms in the fracture healing in T2DOP, in hope of finding novel targets for the treatment of fracture healing in T2DOP.

## 2. Materials and methods

### 2.1 Ethics statement

Animal experiments were approved by the Ethics Committee of The HongQi Hospital of Mudanjiang Medical College and conducted in strict accordance with the *Guide for the Care and Use of Laboratory Animals* published by the Ministry of Science and Technology of the People’s Republic of China in 2006.

### 2.2 Microarray-based gene expression profiling

Type 2 diabetes (T2D)-related dataset GSE95849 [20] (platform: GPL22448) and fracture-related dataset GSE99388 [21] (platform: GPL6246) were retrieved from the Gene Expression Omnibus (GEO) database. The related sample information of the datasets is shown in Supplementary Table 1. The R language ‘limma’ package was used for gene differential analysis, with *p* value < 0.05 as the screening conditions [22]. The GeneCards database was used to predict the genes related to DOP. The jvenn tool was utilized to find the intersecting differentially expressed genes in diabetes mellitus and genes related to DOP. Through the web-based GEne Set AnLysis Toolkit (http://www.webgestalt.org/), Kyoto encyclopedia of genes and genomes (KEGG) enrichment analysis was performed on the signaling pathways that the candidate genes involved. In order to further predict the downstream factors of the key genes, we used the STRING website to search the interaction factors of genes, and the interaction network was visualized using the Cytoscape 3.5.1 software.

### 2.3 Experimental animals

Thirty-two male normal mice (C57BL/6 J) (6–8 weeks old, weighing 20–24 g, specific-pathogen-free, purchased from Huafukang Biotechnology, Beijing, China) and 64 male TLR9 knockout (TLR9^−/−^) mice (C57BL/6 J) (6–8 weeks old, weighing 22–24 g, specific-pathogen-free, purchased from Osaka University, Osaka, Japan) were selected for this study. These mice were randomly assigned into six groups (each n = 16): control (normal mice; Group A), TLR9^−/−^ (TLR9 knockout mice; Group B), T2DOP (STZ induced normal mice; Group C), T2DOP + TLR9^−/−^ (STZ induced TLR9 knockout mice; Group D), T2DOP + TLR9^−/−^ + tumor necrosis factor-α (TNF-α) (STZ induced TLR9 knockout mice; Group E) and T2DOP + TLR9^−/−^ + pyrrolidine dithiocarbamate (PDTC) (STZ induced TLR9 knockout mice; Group F). PDTC (5108–96-3, AbMole) is an inhibitor of the NF-κB signaling pathway, with the injection dose of 50 mg/kg; TNF-α (P6020, Beyotime) is an activator of the NF-κB signaling pathway, with the injection dose of 8 μg/kg [23–25].

The article "Toll-like receptor 9 (TLR9) gene deletion-mediated fracture healing in type II diabetic osteoporosis associates with inhibition of the nuclear factor-kappa B (NF-κB) signaling pathway" was retracted in 2026. Reasons: concerns about the data; concerns about the results or conclusions.

### 2.4 Genotyping of TLR9^−/−^ mice

In order to identify the successful deletion of TLR9 gene in TLR9^−/−^ mice, total RNA was extracted from tail tissues of mice according to the instructions of TRIzol reagents (Life Technologies, Carlsbad, CA), and then was reverse-transcribed into complementary DNA (cDNA). Using reverse transcription quantitative polymerase chain reaction (RT-qPCR) kits, the expression of TLR9 (forward: 5’-GTGCTGAAGGACAGCTCTC-3’; reverse: 5’-GGCGGGTTAGGTTCTGAAAG-3’) was determined with glyceraldehyde-3-phosphate dehydrogenase (GAPDH) serving as a loading control (forward: 5’-CATCACTGCCACCCAGAAGACTG-3’; reverse: 5’-ATGCCAGTGAGCTTCCCGTTCAG-3’) [26].

### 2.5 Establishment of T2DOP mouse models

The T2DOP model was established by 5-day intraperitoneal injection of STZ (40 mg/kg; Sigma-Aldrich, St Louis, MO; prepared with sodium citrate buffer solution [pH 4.5]) into mice in the Group C, Group D, Group E, and Group F. Mice in the Group A and Group B groups were intraperitoneally injected with the same dose of pH 4.5 sodium citrate buffer. After the mice were fasted for 12 h, the glucose level in serum and urine and bone metabolism (serum alkaline phosphatase, serum osteocalcin and serum tartrate resistant acid phosphatase) were measured (Supplementary Table 2). A fasting blood glucose level higher than 11.1 mmol/L indicated successful establishment of T2DOP in mice. After the T2DOP model was successfully prepared, 6 groups of mice were prepared for fracture model construction, and eight mice in each group were randomly selected for indicator determination at 2 and 3 weeks after the fracture model was prepared [27].

### 2.6 Establishment of closed femoral fracture model

A closed femoral fracture model was constructed according to the previously described method [28]. Briefly, 0.2 mL of 0.1% ampicillin was injected subcutaneously into the neck of mice to prevent infection, and 1% pentobarbital (30 mg/kg) was injected intraperitoneally into the mice for anesthesia. After anesthesia, a 10-mm longitudinal skin incision was made on the lateral thigh of mice with ophthalmic scissors to reach the knee joint to expose the femoral intercondylar fossa. A 0.5 mm micro high-speed drill bit was used to drill to reach the upper femoral medullary cavity. Transverse osteotomy was performed in the middle of femoral shaft with a 0.3-mm micro high-speed milling cutter. At the same time, sterile saline was used for local washing and the bones were cooled down to avoid bone necrosis which might result in fracture of the middle femur. The bone chips of the fracture were removed by repeated washing with normal saline. The patella was reset and the joint capsule was sutured. The incision was disinfected with Iodophor and 0.2 mL ampicillin was injected subcutaneously into the back of the mouse neck again.

The article "Toll-like receptor 9 (TLR9) gene deletion-mediated fracture healing in type II diabetic osteoporosis associates with inhibition of the nuclear factor-kappa B (NF-κB) signaling pathway" was retracted in 2026. Reasons: concerns about the data; concerns about the results or conclusions.

### 2.7 Activator and inhibitor of the NF-κB signaling pathway

After the fracture model was successfully established, the mice in Group E were intraperitoneally injected with TNF-α (0.625 mg/mL/kg/day for 3 days; ab141406; Abcam, Cambridge, UK); the mice in Group F were intrathecally injected with PDTC (0.5 μg/10 μL/day; Sigma, GF314) until the end of experimental observation. Mice in Group A, Group B, Group C and Group D were injected with the same dose of normal saline [29,30].

### 2.8 Safranin O staining

Paraffin sections were allowed to stand in a 60°C oven overnight, cleared in xylene I and II solution for 5 min each, rehydrated in 100% alcohol for 2 min, and in 95 and 80% alcohol for 1 min each. The sections were then hydrolyzed with hydrochloric acid ethanol for 1 min, and blued for 3 min. Subsequently, fast green dye solution was dropped into the sections, which were then hydrolyzed with acetic acid solution for 30s. After staining with 1% Safranin O solution for 6 min, the sections were rinsed with 95% alcohol, dehydrated and sealed. Five discontinuous sections in sagittal position were randomly selected from each femoral section. The region of interest (ROI) was defined as 2 mm above/below the fracture line. The images were taken using an Olympus DP80 micro digital camera. The bone tissue, cartilage tissue, fibrous tissue and total callus area in the femoral callus of mice were collected using Image Pro Plus6.0, and the area ratio of the three types of tissues to the total callus area was calculated [31].

### 2.9 Micro-computed tomography (CT)

The ROI of callus was scanned with the micro-CT system (m CT-40, Scanco Medical, Bruttisellen, Switzerland) to analyze the formation of bone tissues in the callus. The measurement range was as follows: 381 layers of axial films were taken from the fracture line, and the callus volume was selected based on two contours in each axial film. The lateral range was the most lateral bone contour of the visible callus, and the internal measurement range was the lateral margin of the femur. Prior to computing the values for each of these outcome measures, a Gaussian filter (sigma = 0.8, support = 1.0) was applied to reduce noise. Subtraction included all mineralized tissues above the threshold (upper threshold 320 HA/ccm, lower threshold 150 HA/ccm) between the two contour lines. The significance of micro-CT parameters was as follows: a) relative volume of trabecular bone: [bone volume/tissue volume (BV/TV)]: the ratio of bone surface area to tissue volume; b) trabecular thickness means the average thickness of phalanx, which is used to describe the structural changes of bone trabecula; trabecular number refers to the number of intersections between bone tissue and non-bone tissue within a given length; trabecular separation indicates the degree of trabecular separation is inversely proportional to the structure of bone tissue in the measured tissue [31].

The article "Toll-like receptor 9 (TLR9) gene deletion-mediated fracture healing in type II diabetic osteoporosis associates with inhibition of the nuclear factor-kappa B (NF-κB) signaling pathway" was retracted in 2026. Reasons: concerns about the data; concerns about the results or conclusions.

### 2.10 Hematoxylin-eosin (HE) staining

Paraffin sections were heated at 55°C for 30 min, then dewaxed three times with xylene (15 min each time), and rehydrated in 100% alcohol and in 95%, 80%, 75% alcohol. Hematoxylin was used to stain the sections for 5 min, which were then washed with deionized water, and observed under a microscope. Following eosin counterstaining for 5 min, the sections were washed with deionized water, and observed under a microscope where the cytoplasm and osteoid were pink. Following 70%, 80%, 95%, 100% alcohol gradient dehydration, 2 min each time, the sections were cleared with xylene, 2 min each time, sealed with neutral resin and observed under a microscope [32].

### 2.11 Western blot assay

The protein expression of femur and surrounding tissues was determined. The tissues were lysed to collect the cells, from the total protein was extracted, with the concentration determined. Next, the protein was separated using electrophoresis and transferred onto membranes. The membrane was then incubated with primary antibodies to GAPDH (1: 1000, ab8245), TLR9 (1: 1000, ab134368), NF-κB (1: 1000, ab32360), tumor necrosis factor receptor-associated factor 6 (TRAF6) (1: 2000, ab33915), p65 (1: 1000, ab32536), caspase-3 (1: 2000, ab184787), and bone morphogenetic protein 7 (BMP7) (1: 1000, ab129156) and then with secondary antibody (1: 2000, ab205719 or 205,718). All the aforementioned antibodies were purchased from Abcam. The gray value of the bands was analyzed by Image J software after development with enhanced chemiluminescence [33].

The article "Toll-like receptor 9 (TLR9) gene deletion-mediated fracture healing in type II diabetic osteoporosis associates with inhibition of the nuclear factor-kappa B (NF-κB) signaling pathway" was retracted in 2026. Reasons: concerns about the data; concerns about the results or conclusions.

### 2.12 Statistical analysis

All data obtained from three independent experiments were expressed as mean ± standard deviation and analyzed by SPSS 26.0 statistical software (IBM Corp., Armonk, NY). The statistical significance was measured using independent sample *t*-test (two-group data), one-way analysis of variance (ANOVA) (multi-group data) with Tukey’s post hoc test or repeated measures ANOVA (multi-group data at different time points) with Bonferroni’s post hoc test. A value of *p* < 0.05 was statistically significant.

## 3. Results

### 3.1 Bioinformatics analysis indicates that TLR9 may affect T2DOP by mediating the NF-κB signaling pathway

T2DOP is a common complication of T2D with an increasing incidence over the past few decades [2], leading to increased fracture risk and impaired bone healing [3]. TLR9, as one of the most important TLR protein family, has been found to be significantly highly expressed in hip fracture rats [11]. Interestingly, TLR9 deficiency was found to enhance glucose tolerance and improve insulin sensitivity in T1DM [34]. Therefore, we explored the effect of TLR9 on T2DOP (Supplementary Figure 1).

In order to explore the important regulatory factors involved in T2DOP, we firstly performed differential analysis of the T2D-related dataset GSE95849. A total of 2051 differentially expressed genes were screened, comprised of 1273 significantly upregulated genes and 778 downregulated genes (Figure 1a). In addition, 624 genes related to DOP were identified from the GeneCards database, and 54 candidate genes were obtained following intersection analysis of the significantly highly expressed genes in T2D and DOP-related genes (Figure 1b). The results of KEGG enrichment analysis of the 54 candidate genes using WEB-based GEne SeT AnaLysis Toolkit revealed that these genes were mainly involved in TLR signaling pathway, TNF signaling pathway, IL-17 signaling pathway and AGE-RAGE signaling pathway (Figure 1c), with the TLR signaling pathway more prominent (Figure 1d). Meanwhile, 13 genes were involved in the TLR signaling pathway (Figure 1d). Additionally, differential analysis of the fracture-related dataset GSE99388 demonstrated that TLR9 showed lower expression in the fracture healing samples than that in fracture samples (Figure 1e). Moreover, TLR9 expression was notably higher in T2D samples than that in control samples after differential analysis of the T2D-related dataset GSE95849 (figure 1f). Therefore, we predicted that TLR9 was significantly overexpressed in T2DOP.

**Figure 1.** Bioinformatics analysis to predict the differential genes and their molecular interactions in T2DOP. A, A volcano map for differentially expressed genes in T2D samples in the T2D-related dataset GSE95849. The X-axis indicates -log10 (*p* value), and the Y-axis indicates logFC. B, Venn map of significantly highly expressed genes in T2D and DOP-related genes. C, KEGG enrichment analysis of the 54 candidate genes. D, Venn map for the intersection of genes involved in signaling pathway and total gene set. E, The expression of TLR9 in the fracture healing samples (n = 30) and fracture samples (n = 11) in the fracture-related dataset GSE99388. F, TLR9 expression in T2D samples (n = 6) and control samples (n = 6) in the T2D-related dataset GSE95849. G, The interaction network of TLR9 gene. H, KEGG enrichment analysis of TLR9 interaction factor pathways.

The article "Toll-like receptor 9 (TLR9) gene deletion-mediated fracture healing in type II diabetic osteoporosis associates with inhibition of the nuclear factor-kappa B (NF-κB) signaling pathway" was retracted in 2026. Reasons: concerns about the data; concerns about the results or conclusions.

In order to further predict the downstream pathway of TLR9, we plotted an interaction network of the TLR9 gene through the STRING website (Figure 1g). Further KEGG enrichment analysis of these interaction factors showed that genes were mainly concentrated in the NF-κB signaling pathway (Figure 1h). Published literature has reported that TLR9 can regulate the NF-κB signaling pathway [35], which may be related to the occurrence of T2DOP [18].

Overall, the above results suggest that TLR9 may affect T2DOP by mediating the NF-κB signaling pathway.

### 3.2 TLR9 knockout promotes the regeneration of bone tissues and cartilage area in the callus, and reduces the area of fibrous tissues in T2DOP mice

Subsequently, we moved to further explore the effect of TLR9 on T2DOP. Safranin O staining results shown in Figure 2a suggested that 3 weeks after fracture, trabeculae of new bone was obvious in Group A and Group B, cartilage osteogenesis was active, braided bone replaced the original cartilage tissue, and visible bone connection was formed at fracture ends, especially in Group B. In Group C, there were still a lot of fibrous tissues and undifferentiated mesenchymal tissues in the callus, a small amount of braided bone was formed, and no bone connection was formed at the fracture end of right femur fracture. In Group D, there was obvious cartilage tissue formation, cartilage osteogenic process and bone trabecula formation, with obvious bone connection formed on the fracture end.

**Figure 2.** TLR9 knockout promotes the regeneration of bone tissues and cartilage area in the callus, and reduces the area of fibrous tissues in T2DOP mice. The mice were randomly assigned into following groups: control (normal mice; Group A), TLR9^−/−^ (TLR9 knockout mice; Group B), T2DOP (STZ induced normal mice; Group C), and T2DOP + TLR9^−/−^ (STZ induced TLR9 knockout mice; Group D). A, Safranin O staining for histological observation of femoral callus in mice with different treatment at the 3^rd^ week. B, Safranin O staining for histological observation of and qualification for bony cartilage area of femoral callus in mice with different treatment. C, Safranin O staining for histological observation of and qualification for cartilaginous area of femoral callus in mice with different treatment. D, Safranin O staining for histological observation of and qualification for fibrous callus area of femoral callus in mice with different treatment. E, RT-qPCR and Western blot assay were used to verify the knockout efficiency of TLR9 in Group B. * *p* < 0.05 *vs*. Group A. ^#^ *p* < 0.05 *vs*. Group C. The measurement data were expressed as mean ± standard deviation. The comparison among multiple groups at different time points was conducted by repeated measures ANOVA, followed by Bonferroni’s post hoc test. n = 16.

The article "Toll-like receptor 9 (TLR9) gene deletion-mediated fracture healing in type II diabetic osteoporosis associates with inhibition of the nuclear factor-kappa B (NF-κB) signaling pathway" was retracted in 2026. Reasons: concerns about the data; concerns about the results or conclusions.

Based on the measurement results of the three kinds of tissues in the callus (Figure 2b-d), after 2 weeks of fracture modeling, compared with Group A, the areas of bone tissues and cartilage in the callus of Group C were markedly decreased, and the area of fibrous tissues was significantly increased; the areas of bone tissues and cartilage in the callus of Group B were notably increased, and the area of fibrous tissues was significantly decreased. Compared with Group C mice, Group D mice had notably increased areas of bone tissues and cartilage in the callus, and significantly decreased area of fibrous tissues. Further, we performed RT-qPCR and Western blot assay to verify the knockout efficiency of TLR9 in the Group B where TLR9 showed no expression (Figure 2e), suggesting that TLR9^−/^ mice were successfully constructed.

Together, these results suggest that deficiency of TLR9 can promote the regeneration of bone tissues and cartilage area in the callus, and reduce the area of fibrous tissues in T2DOP mice.

### 3.3 TLR9 knockout promotes fracture recovery in T2DOP mice

Furthermore, we aimed to elucidate the impact of TLR9 knockout on bone recovery after injury. We used micro-CT to measure the changes in BMD, BV/TV, connectivity density, trabecular number, trabecular separation, and trabecular thickness after different treatment. The results (Figure 3a-f) revealed that relative to Group A, Group C had markedly lower BMD, BV/TV, connectivity density and trabecular number, and notably increased trabecular separation, while the trabecular thickness was not significantly changed; Group B had markedly increased BMD, BV/TV, connectivity density and trabecular number, and notably reduced trabecular separation, without significant changes in trabecular thickness. Compared with Group C, BMD, BV/TV, connectivity density and trabecular number were significantly increased, while the trabecular separation was markedly decreased, and the trabecular thickness was not significantly changed in Group D.

The article "Toll-like receptor 9 (TLR9) gene deletion-mediated fracture healing in type II diabetic osteoporosis associates with inhibition of the nuclear factor-kappa B (NF-κB) signaling pathway" was retracted in 2026. Reasons: concerns about the data; concerns about the results or conclusions.

**Figure 3.** TLR9 knockout facilitates fracture recovery in T2DOP mice. The mice were randomly assigned into following groups: control (normal mice; Group A), TLR9^−/−^ (TLR9 knockout mice; Group B), T2DOP (STZ induced normal mice; Group C), and T2DOP + TLR9^−/−^ (STZ induced TLR9 knockout mice; Group D). A, Quantitative analysis for the change of BMD in mice with different treatment. B, Quantitative analysis for the change of BV/TV in mice with different treatment. C, Quantitative analysis for the change of connectivity density in mice with different treatment. D, Quantitative analysis for the change of trabecular number in mice with different treatment. E, Quantitative analysis for the change of trabecular separation in mice with different treatment. F, Quantitative analysis for the change of trabecular thickness in mice with different treatment. * *p* < 0.05 *vs*. Group A. ^#^ *p* < 0.05 *vs*. Group C. The measurement data were expressed as mean ± standard deviation. The comparison among multiple groups at different time points was conducted by repeated measures ANOVA, followed by Bonferroni’s post hoc test. n = 16.

The above results suggest that TLR9 can slow fracture recovery, while TLR9 knockdown promotes fracture recovery.

### 3.4 TLR9 knockout enhances fracture healing and increases callus transformation rate in T2DOP mice

The effect of TLR9 knockout on the fracture healing was the next focus of our study. Based on the results of HE staining (Figure 4), most of the fracture ends in Group A and Group B showed bony union, along with continuous callus around the broken ends. Most of the callus was bony callus, with a small number of chondrocytes but no cartilage Island. The trabeculae were uniform in thickness and arranged in order, with high maturity and obvious lamellar bone formation. In Group C, there were a large number of chondrocytes between the fracture ends; cartilage Island was visible; the number of bone trabeculae was small, with low maturity; the arrangement of trabeculae was in disorder, and the spacing was wide; most of the callus was bony callus. In Group D mice, the fracture ends partially healed, and continuous callus passed around the fracture ends; in the callus, bony callus and cartilaginous callus co-existed; chondrocytes existed but no cartilage Island was found; trabeculae was relatively mature and arranged orderly, and a small amount of lamellar bone formation was seen. Compared with the Group C, Group D mice displayed accelerated fracture healing process and transformation rate from cartilage callus to bony callus in T2DOP mice.

The article "Toll-like receptor 9 (TLR9) gene deletion-mediated fracture healing in type II diabetic osteoporosis associates with inhibition of the nuclear factor-kappa B (NF-κB) signaling pathway" was retracted in 2026. Reasons: concerns about the data; concerns about the results or conclusions.

**Figure 4.** TLR9 knockout accelerates fracture healing and callus transformation rate in T2DOP mice. HE staining for new bones at the 3^rd^ week in mice with different treatment. The mice were randomly assigned into following groups: control (normal mice; Group A), TLR9^−/−^ (TLR9 knockout mice; Group B), T2DOP (STZ induced normal mice; Group C), and T2DOP + TLR9^−/−^ (STZ induced TLR9 knockout mice; Group D). * indicates lesion area. n = 16.

Altogether, these data reveal that TLR9 knockout can increase fracture healing and callus transformation rate in T2DOP mice.

### 3.5 TLR9 knockout inhibits the NF-κB signaling pathway in T2DOP mice

It has been reported that TLR9 can regulate the NF-κB signaling pathway [35], which may be related to the occurrence of T2DOP [18]. These lines of evidence allowed us to speculate whether TLR9 affected femoral fracture through the NF-κB signaling pathway.

Western blot assay results showed that there was no TLR9 protein expression in Group B and Group D (Figure 5a, b). Compared with Group A, Group B showed a decline in the protein expression of TRAF6, NF-κB, p65 and caspase-3, and an increase in the expression of BMP-7; Group C displayed significantly increased protein expression of TRAF6, NF-κB, p65 and caspase-3, and markedly decreased expression of BMP-7. Relative to Group C, Group D had notably increased protein expression of TRAF6, NF-κB, p65 and caspase-3, accompanied by increased expression of BMP-7.

**Figure 5.** TLR9 knockout inhibits the NF-κB signaling pathway in T2DOP mice. The mice were randomly assigned into following groups: control (normal mice; Group A), TLR9^−/−^ (TLR9 knockout mice; Group B), T2DOP (STZ induced normal mice; Group C), and T2DOP + TLR9^−/−^ (STZ induced TLR9 knockout mice; Group D). A, The expression of TLR9 and NF-κB signaling pathway related proteins in the femoral fracture end tissues of mice with different treatment as determined by Western blot assay. B, Quantitative analysis of panel A. * *p* < 0.05 *vs*. Group A. ^#^ *p* < 0.05 *vs*. Group C. The measurement data were expressed as mean ± standard deviation. The comparison among multiple groups was performed by one-way ANOVA, followed by Tukey’s post hoc test. n = 16.

These results suggest that TLR9 knockout can inhibit the NF-κB signaling pathway in T2DOP mice.

### 3.6 TLR9 knockout promotes fracture healing in T2DOP by inhibiting the NF-κB signaling pathway

Finally, we sought to characterize the effect of TLR9 regulating the NF-κB signaling pathway on fracture healing in T2DOP. Safranin O staining results (Figure 6a) demonstrated that compared with Group D, the areas of bone tissues and cartilage in the callus of Group E were decreased and fibrous tissue area increased, while Group F displayed opposite results. The results of micro-CT (Figure 6b-g, Supplementary Figure 2) revealed that in comparison to Group D, Group E had marked declines in regard to BMD, BV/TV, connectivity density, and trabecular number, increased trabecular separation and unchanged trabecular thickness; while Group F had significant increases in the BMD, BV/TV, connectivity density, and trabecular number, a decline in the trabecular separation and no changes in the trabecular thickness.

The article "Toll-like receptor 9 (TLR9) gene deletion-mediated fracture healing in type II diabetic osteoporosis associates with inhibition of the nuclear factor-kappa B (NF-κB) signaling pathway" was retracted in 2026. Reasons: concerns about the data; concerns about the results or conclusions.

**Figure 6.** TLR9 knockout promotes the fracture healing in T2DOP mice through NF-κB signaling pathway inactivation. The mice were randomly assigned into following groups: T2DOP + TLR9^−/−^ (STZ induced TLR9 knockout mice; Group D), T2DOP + TLR9^−/−^ + TNF-α (STZ induced TLR9 knockout mice; Group E) and T2DOP + TLR9^−/−^ + PDTC (STZ induced TLR9 knockout mice; Group F). A, Safranin O staining for quantification for bony cartilage area, cartilaginous area and fibrous callus area of femoral callus in mice with different treatment. B, Quantitative analysis for the change of BMD in mice with different treatment. C, Quantitative analysis for the change of BV/TV in mice with different treatment. D, Quantitative analysis for the change of connectivity density in mice with different treatment. E, Quantitative analysis for the change of trabecular number in mice with different treatment. F, Quantitative analysis for the change of trabecular separation in mice with different treatment. G, Quantitative analysis for the change of trabecular thickness in mice with different treatment. H, The expression of TLR9 and NF-κB signaling pathway related proteins in the femoral fracture end tissues of mice with different treatment determined by Western blot assay. * *p* < 0.05 *vs*. Group D. The measurement data were expressed as mean ± standard deviation. The comparison among multiple groups was performed by one-way ANOVA, followed by Tukey’s post hoc test, and that among multiple groups at different time points by repeated measures ANOVA, followed by Bonferroni’s post hoc test. n = 16.

Western blot assay (Figure 6h) results revealed that compared with Group D, Group E showed a marked increase in the protein expression of TRAF6, NF-κB, p65 and caspase-3, as well as a decline in the expression of BMP-7; Group F displayed significantly decreased protein expression of TRAF6, NF-κB, p65 and caspase-3, and increased expression of BMP-7.

Overall, TLR9 knockout can promote fracture healing by inhibiting the NF-κB signaling pathway in T2DOP mice.

The article "Toll-like receptor 9 (TLR9) gene deletion-mediated fracture healing in type II diabetic osteoporosis associates with inhibition of the nuclear factor-kappa B (NF-κB) signaling pathway" was retracted in 2026. Reasons: concerns about the data; concerns about the results or conclusions.

## 4. Discussion

DOP is regarded as a serious and chronic complication of diabetes occurring at the bone and joint sites, the pathogenesis of which is still in requirement of further exploration [36]. Of note, in order to seek optimal fracture prevention for patients with DOP, it is requisite to conduct further assessment of the efficacy of osteoporosis therapies in the setting of diabetes [37]. In the present study, we set out to explore the role of TLR9 and the NF-κB signaling pathway in T2DOP. The results unfolded that TLR9 depletion-mediated NF-κB signaling pathway inactivation could promote the fracture healing in T2DOP.

In the first place, this study revealed that knockout of TLR9 promoted the fracture healing of T2DOP mice, which is reflected not only by the facilitated regeneration of bone tissue and cartilage area in the callus and reduced area of fibrous tissues, but also the changed BMD, BV/TV, connectivity density, trabecular number, trabecular separation and trabecular thickness, and improved bone morphology and structure in T2DOP mice. Similar with our findings, the participation of TLR9 in diabetes or bone-related diseases has been reported; for instance, the downregulation of TLR9 due to Dkk-1 knockdown contributed to alleviated cartilage destruction as well as subchondral bone injury in osteoarthritic knee joints, in part by modulating the bone density [38]. Moreover, the TLR-4/TLR-9/NF-κB signaling pathway upregulated by neutrophils release extracellular traps triggers NLRP3 inflammasome activation to sustain inflammation in the diabetic wound [39]. In addition, Gan et. al. identified that TLR9 and NF-κB p65 were upregulated in rats with lung injury in the presence of hip fracture [11]. Overall, these previous studies could support our findings regarding the alleviatory role of knockout of TLR9 in T2DOP.

Importantly, we further extended the mechanistic exploration on the effect of TLR9 on T2DOP, and found that TLR9 could inhibit the activation of the NF-κB signaling pathway in T2DOP. Intriguingly, the promoting role of the NF-κB signaling pathway in the progression of DOP has been highlighted by many studies over the past decade; specifically, the inhibited activity of the NF-κB signaling pathway achieved by knockdown of cereblon could contribute to alleviation in receptor activator of NF-κB ligand-induced osteoclastogenesis, thereby protecting against DOP induced by STZ in a mouse model [40]. Besides, the repressed activation of the NF-κB signaling pathway by Bergapten could protect trabecular structure and reduce osteoclastogenic differentiation, thereby inhibiting DOP [41]. To date, a large number of previous studies have discovered the regulatory relationship between TLR9 and NF-κB in multiple diseases. For instance, partially in consistency with our result, it was revealed that TLR9 could lead to the activation of NF-κB during murine herpesvirus 68 reactivation [42]. In addition, Gomes et al. demonstrated that TLR9 is essential for MAPK/NF-κB activation in a manner independent of TLR2 or TLR6, which triggered host resistance to Brucella abortus [43]. As previously reported, TLR9, in combination with BCR as well as mutant isoforms of MYD88, could result in sustained activity of NF-κB in the activated B-cell-like subtype of diffuse large B-cell lymphoma [44]. Furthermore, Nishimoto et al. have confirmed that genetic deletion of TLR9 brings about suppression in the activation of NF-κB activation in ischemic muscle [45]. Therefore, it is concluded in this mechanistic exploration that the inhibitory role of knockout of TLR9 in T2DOP is achieved by the downregulation of the NF-κB signaling pathway.

The article "Toll-like receptor 9 (TLR9) gene deletion-mediated fracture healing in type II diabetic osteoporosis associates with inhibition of the nuclear factor-kappa B (NF-κB) signaling pathway" was retracted in 2026. Reasons: concerns about the data; concerns about the results or conclusions.

## 5. Conclusion

The current study demonstrated that knockout of TLR9 could promote fracture healing in T2DOP *via* suppression of the NF-κB signaling pathway (Figure 7). This finding may provide a potential direction for the treatment of T2DOP. However, the specific mechanism regarding the role of the NF-κB signaling pathway in T2DOP requires further investigation. Moreover, the clinical feasibility of TLR9-targeted therapy for the treatment of T2DOP still warrants further validation.

**Figure 7.** The mechanism graph of the regulatory network and function of TLR9. Knockout of TLR9 promotes fracture healing in T2DOP *via* suppression of the NF-κB signaling pathway.

### Limitaion

However, the present results that the TLR9/NF-κB regulatory axis played an important role in the pathogenesis of T2DOP were mainly based on the mouse T2DOP model, and thus whether the TLR9/NF-κB regulatory axis functions consistently in clinical patients with T2DOP still needs further verification. In addition, TLR9/NF-κB mediated inflammation plays a role in the pathogenesis of T2DOP is worthy of further exploration, because inflammation itself is closely related to diabetes and bone diseases, such as arthritis.

## Supplementary Material

Supplemental Material
